The article "Hybrid Approach Named HUAPO Technique to Guide the Lander Based on the Landing Trajectory Generation for Unmanned Lunar Mission" was published in 2022. Journal: Comput Intell Neurosci.

# Hybrid Approach Named HUAPO Technique to Guide the Lander Based on the Landing Trajectory Generation for Unmanned Lunar Mission

**DOI:** 10.1155/2022/4698936

**Published:** 2022-06-07

**Authors:** Shaikh Abdul Latif, Ibrahim M. Mehedi, Ahmed I. M. Iskanderani, Mahendiran T. Vellingiri, Rahtul Jannat

**Affiliations:** ^1^Department of Nuclear Engineering, King Abdulaziz University, Jeddah, Saudi Arabia; ^2^Center of Research Excellence in Intelligent Engineering Systems (CEIES), King Abdulaziz University, Jeddah 21589, Saudi Arabia; ^3^Department of Electrical and Computer Engineering (ECE), King Abdulaziz University, Jeddah 21589, Saudi Arabia; ^4^Department of Electrical & Electronic Engineering (EEE), BRAC University, Dhaka, Bangladesh

## Abstract

This manuscript proposes a hybrid method for landing trajectory generation of unmanned lunar mission. The proposed hybrid control scheme is the joint execution of the human urbanization algorithm (HUA) and political optimizer (PO) with radial basis functional neural network (RBFNN); hence it is named as HUA-PORFNN method. The HUA is a metaheuristic method, and it is used to solve several optimization issues and several nature-inspired methods to enhance the convergence speed with quality. On the other hand, multiple-phased political processes inspire the PO. The work aims to guide the lander with minimal fuel consumption from the initial to the final stage, thus minimizing the lunar soft landing issues based on the given cost of operation. Here, the HUAPO method is implemented to overcome thrust discontinuities, checkpoint constraints are suggested for connecting multi-landing phases, angular attitude rate is modeled to obtain radical change rid, and safeguards are enforced to deflect collision along with obstacles. Moreover, first, the issues have been resolved according to the proposed HUAPO method. Here, energy trajectories with 3 terminal processes are deemed. Additionally, the proposed HUAPO method is executed on MATLAB/Simulink site, and the performance of the proposed method is compared with other methods.

## 1. Introduction

The moon is the adjacent celestial body to the earth that moderates the wobble of earth on its axis, leading to a relatively standard climate for billions of years. Only one face of the moon is visible when viewed from earth because the moon rotates on its axis at a similar speed as it orbits the earth (it is in a coherent cycle with the earth). In 1959, the Soviet Union's unscrewed Luna 1 and II firstly landed on the moon, and in April 2019, 7 nations followed. The USA sent 3 groups of robotic missions to explore the possibility of human landing on the moon: (i) for taking lunar surface imagery, the Rangers (1961–1965) were designed, and they sent those imageries to earth until the spacecraft is shattered; (ii) Lunar Orbiters (1966–1967) mapped the surface to detect the sites of landing; (iii) Surveyors (1966–1968) aim was demonstrating the feasibility of soft landings. Recently, space researchers have become increasingly focused on exploring the moon because the moon is more metallic than imagined by scientists. For example, helium-3 is plentiful on the moon; it is employed in nuclear fusion. Also, it may be a future energy source. The Lunar Reconnaissance Orbiter ensured the presence of iron and titanium oxides under the moon's surface. The moon is a pioneering site for research on other planets [1, 2]. As for the feasible advantages of lunar research, the Indians, Americans, Japanese, Europeans, and Chinese scientists plan to go back to the moon [3]. NASA officially did not launch new lunar programs after undertaking the Apollo program 1961–1972. After a long hiatus, the US robotic missions resumed lunar exploration in the 1990s by Clementine together with lunar Prospector. These two missions showed that there might be water ice at the lunar poles, but the Prospector spacecraft did not prove the evidence of significant water. In 2009, the USA launched a novel series of robotic missions and the combined launch of NASA's Lunar Reconnaissance Orbiter (LRO), Lunar Crater Observation including sensing satellite. In this, Lunar Crater Observation, including sensing satellite, has confirmed the existence of water on the moon. NASA recently launched a Lunar CATALYST program formulated to aid and incentivize private companies involved in lunar research [4–6].

The article "Hybrid Approach Named HUAPO Technique to Guide the Lander Based on the Landing Trajectory Generation for Unmanned Lunar Mission" was published in 2022. Journal: Comput Intell Neurosci.

The lunar soft landing (LSL) is a challenging task of lunar exploration, where the lunar module lands smoothly on the lunar surface using a reversal propeller force [7]. This study proposes to acquire a fuel-optimum path of LSL with variable propulsion. This trajectory optimization (TO) issue is designed into constrained optimum control complexity linked to key features of the problem [8–12]. The Japanese lunar exploration plan is a robot and human travel program for the moon; its principal purpose is to clarify the origin and the moon's evolution and its future use for the moon [13–16].

The most crucial strategy of lunar exploration is soft landing, and also it is essential for lunar research in the above-represented countries [17]. However, the security, precision, cost, and proficiency are the significant deficiencies of lunar soft landing missions. The probes on TO for LSL are efficiently contributed to enhancing such deficiencies [18]. In 2018, China planned to make a soft landing on the back of the moon [19]. However, unfortunately, the mission was a failure. The moon's hemisphere is called the back of the moon, which is distant from the earth; also, it is protected by radio transmissions coming from the earth.

The article "Hybrid Approach Named HUAPO Technique to Guide the Lander Based on the Landing Trajectory Generation for Unmanned Lunar Mission" was published in 2022. Journal: Comput Intell Neurosci.

Furthermore, the far-side terrain is rugged. In this situation, India launched the Vikram lander on July 22, 2019, for a soft landing on the back of the moon; if it succeeds in that effort, India will have pride in being the first country to send there. The purpose of this lander is to descend toward and comes to rest on the astronomical body's surface, and the lander forms a soft landing; after that, the probe operates [20]. This manuscript proposes a hybrid method for landing trajectory generation of unmanned lunar mission. The proposed hybrid control scheme is the joint execution of the human urbanization algorithm (HUA) and political optimizer (PO) with radial basis functional neural network (RBFNN). Hence, it is named as HUA-PORFNN method. The remaining segment of this manuscript is designed as follows: Segment 2 describes the recent investigation works with its background. Segment 3 explains the multi-phase problem formulation for a lunar landing. Segment 4 illustrates the proposed HUA-PORFNN approach. Segment 5 demonstrates the simulation result and discussion of HUA-PORFNN and existing approaches. Finally, Segment 6 concludes the manuscript.

## 2. Recent Research Work: A Brief Review

Several research works previously existed in literature based on landing trajectory generation and energy optimization of uncrewed lunar mission with numerous methods and features. Specific works are reviewed here.

Qu [21] has suggested an incorporated trajectory optimization system with the initialization modes for a soft lunar landing. Here, the two essential missions of the Apollo spacecraft were (i) Landing from less lunar orbit and (ii) Vertical Takeoff Vertical Landing (VTVL) (promising mobility type) on the lunar surface. Path optimization was defined as obstacles caused through uninterrupted thrust, multiple phase relations, tab of the approach angle, and avoidance of obstacles. The R-function was used to overcome the discontinuities of thrust. The checkpoint controls were established to link multi-landing stages. The approach angle ratio was formulated to avoid radical changes, and safety rules were undertaken to avoid collisions with obstacles. As a result, the emotional issues were typical with problem restraints. The unified system depends on Gauss pseudospectral method (GPM) with a nonlinear programming solver tailored to address the issues proficiently. Ma et al. [22] have presented the issue of fuel-optimum lunar soft landing path optimization with the help of variable thrust propulsion. Here, (i) the lunar soft landing TO issue was framed with 3-D kinematics, dynamics models, boundary levels, and strictly described path controls. Then, the TO problem designed using the simultaneous dynamic optimization method was solved. The optimum control solutions commonly contain a thrust profile named “bang-bang,” as there were limits to the amount of engine thrust. There was a problem dealing with breakpoints on control profiles in the general simultaneous dynamic optimization method. Here, the innovative adaptive mesh refinement technique depending on the standard Hamiltonian profile was suggested to solve the problem of finding gaps in the thrust profile. Mathavaraj et al. [13] have introduced a multiple phase constrained fuel-optimal trajectory design method depending on Legendre pseudospectral philosophy. Here, the aim was to recognize the optimum method to successfully navigate the lunar lander from perilune (18 km altitude) to transfer orbit 100 m altitude on a particular landing site. After reaching an altitude of 100 meters, there was a task complex re-target phase, which contains various goals, so it was not considered in this study. The introduced system considers different mission barriers from perilune to landing location at many phases. Such barriers involve phase-1: from 18 km–7 km altitude, navigation accuracy was wretched, phase-2: holding the lander attitude for 35 sec via view camera execution to get the navigation fault, and phase-3: over the landing location, the accuracy of navigation was excellent.

The article "Hybrid Approach Named HUAPO Technique to Guide the Lander Based on the Landing Trajectory Generation for Unmanned Lunar Mission" was published in 2022. Journal: Comput Intell Neurosci.

Ma et al. [23] have suggested a trajectory optimization system for lunar rovers that performs VTVL using variable thrust propulsion in terrain. (i) A TO problem of VTVL including 3-D kinematics with dynamics mode, boundary stages, and trajectory constraints was designed. Moreover, a finite-element model transcribes the designed TO problem as nonlinear programming complexity addressed through an exceedingly proficient nonlinear programming solver. A backtracking approach depending on homotopy was used to improve integration in solving the TO problem of VTVL. Mehedi et al. [24] have suggested to increase lunar landing efficiency, considering the sole probe positioned usage in auxiliary orbit around the moon, based on mission costs, trajectory, and visibility. For this purpose, two semicircular orbits classified by the constant behavior of the half-key axis, peculiarity, and inclination were suggested. In addition, the possibilities for gaining continuous communication with the earth's ground stations and landers were explored, along with the advantages of exploring the lander's position and velocity. Riu et al. [25] have presented a small-scale mission conception to classify the perpetually shaded areas of the lunar South Pole. For the first time, MARAUDERS targets to measure the presence, distribution, and instability in the perpetually shaded crater, using 12 sorted impacts over existing orbital measurements. A total of 15 permanently shaded areas were classified as the candidates for a landing site for surveys. The scientific principle depended on the penetrometer, which has proven to be a proficient method for estimating the properties of regolith from acceleration profiles. Here, this conception was demonstrated by simulating the surface interactions amid the probes and lunar regolith. Thus, deceleration profiles clarify data about the main regolith features and then assist in distinguishing between the two ice-regolith end members. Mehedi and Islam [26] have presented the fuel-optimum TO problem of LSL with the help of variable thrust propulsion. Here, the TO problem of soft lunar landing along with 3-D kinematics and dynamics, and the constraints of boundary and trajectory were described. Simultaneously, the TO problem designed through dynamic optimization strategy is solved.

The article "Hybrid Approach Named HUAPO Technique to Guide the Lander Based on the Landing Trajectory Generation for Unmanned Lunar Mission" was published in 2022. Journal: Comput Intell Neurosci.

### 2.1. Background of the Research Work

The recent research work review represents the landing trajectory generation, and energy optimization of unmanned lunar mission is a significant contributing factor. Here, this problem is solved in a single step with the help of the point mass method denoting the lander craft. The lunar landing has solved the problem of single level determining only some mission impediments. However, solving the landing issue as a phase is not realistic. The spaceship is to be effected only through propulsive and solar gravitational force. Therefore, the optical controller must calculate the camera sensor processing time and its fundamental approach in the practical situation. As nonlinear terms use a homotopy-iterative model instead of linearization, no reference trajectory is required, and convex optimization regains early-guess freedom. This control program is represented as the DNN-based approach.

Moreover, concerning the fuel optimization issue, the DNN-based model is, in some instances, difficult to integrate. The homotopy model is utilized for solving this issue and acquires the fuel optimization issues, and the solutions initializing from DNN forecasted solutions for the issues of optimum energy. The design of optical control is illustrated with this additional constraint and a soft landing constraint. Only the terminal stage of the lander issue is deemed with the de-orbit phase, and then the transfer orbit phase is resolved appropriately. The two-dimensional is defined as a motion equation using optimal control design. Through optimal control creation, all mission barriers are designed and incorporated into the design. These drawbacks mentioned above inspired to do this research work.

The article "Hybrid Approach Named HUAPO Technique to Guide the Lander Based on the Landing Trajectory Generation for Unmanned Lunar Mission" was published in 2022. Journal: Comput Intell Neurosci.

## 3. Multi-Phase Problem Formulation for Lunar Landing

First, starting the trajectory from the circular parking orbit, the spacecraft is to be de-boosted from 100 km to 18 km altitude, as shown in Figure 1. Then, the lander is inserted into the equipped descent phase at the orbit height of 18 km. The propellant engines are turned on closer to the phase, and in a dominated manner, the lander velocity is diminished to allow it to soft-land on the lunar surface. For landing the lunar module onto the lunar surface, there are three types of phases transformed that are needed to be accomplished. They are (i) de-orbit maneuver, (ii) transfer orbit or coasting, and (iii) powered descent. Based on the Hohmann transfer process for entering an 18 km attitude, the de-orbit phase is to operate the lander from a 100 km parking orbit. From the transfer orbit phase, the lander is configured to coast to 18 km, based on the suitable process while decelerating to the lander for accessing the landing site. The rapid and out-of-plane maneuver is minutely planned based on the extra fuel consumption cost which is eliminated.

### 3.1. System Dynamics of the Lunar Landing

It must specify a proper synchronized system in the inertial center frame of the moon to define the motion of the lander and evaluate the equations of motion due to the physical laws which regulate the system. The 3-dimensional motion equations and rotational velocity of the moon are evaluated based on the vehicle as a point mass in the lunar gravity field, which is expressed as follows:

(1) $$\begin{array}{c} R=W,\\ \theta =\frac{U}{R\;\cos\;\phi },\\ \phi =\frac{U}{R},\\ W=\frac{t\text{Sin}\beta }{M}-\frac{\mu }{R^{2}}+\frac{\left(U^{2}+U^{2}\right)}{R}+\left(-2U\omega \text{Cos}\phi +R\omega^{2}{\text{Cos}}^{2}\phi \right). \end{array}$$

Here, from the center of the moon, the radial distance is denoted as *r* and *h*, and *U,* V, and *W* are expressed as the latitude and longitude traced by the lander elements of tangential, across, and vertical velocity. The immediate mass of the lander is denoted as m. Finally, the particular impulse of the engine is represented as *Isp*.

(2) $$\begin{array}{c} U=\frac{\left(t\text{Cos }x\text{ Cos }\beta \right)}{M}+\frac{\left(-UW+UV\text{ Tan}\phi \right)}{R}\\ +\left(-2W\omega \text{Sin}\phi +2V\omega \text{Sin}\phi \right),\\ V=\frac{\left(t\text{Sin }x\text{ Cos }\beta \right)}{M}+\frac{\left(-UW-U^{2}\text{ Tan}\phi \right)}{R}\\ +\left(-2U\omega \text{Sin}\phi -R\omega^{2}\text{Sin}\phi \text{Cos}\phi \right),\\ M=-\frac{t}{i_{SP}G}. \end{array}$$

The standardization is necessary for the numerical preparation of the variables in the optimization process. Additionally, from the center of the moon, the factors which are utilized, such as initial distance of lander (ri), radius of the moon (rm), and initial mass of lander's (mi), and the equations for the factors are expressed as follows:

(3) $$\begin{array}{c} v_{N}=\left|\sqrt{\frac{\mu }{R_{i}}}\right|,\\ D_{N}=\left|R_{M}\right|,\\ M_{N}=\left|M_{i}\right|. \end{array}$$

The article "Hybrid Approach Named HUAPO Technique to Guide the Lander Based on the Landing Trajectory Generation for Unmanned Lunar Mission" was published in 2022. Journal: Comput Intell Neurosci.

### 3.2. Selection of Cost Function

The fuel consumption of spacecraft is to be diminished for explorations of useful lunar to carry an enlarged payload mass. So for the issues of optimal control, the cost function is chosen as a reduction of acceleration.

(4) $$\begin{array}{c} j=\int_{T_{0}}^{T_{f}}\frac{t}{M}\text{ d}t. \end{array}$$

### 3.3. Lunar Landing

A typical structure of a lunar lander is shown in Figure 2. Numerically, the issues of lunar descent have been corrected, which is an overall incorporated approach. The conventional solution, dissimilar from the suitable method, moreover bears several restrictions: the lunar surface is regarded as a plane surface, and the conditions of centrifugal acceleration are not comprised. Among the equation of motion, the conventional solution can be considerably enhanced by evaluating a standard spherical lunar surface involving the conditions of centrifugal acceleration.

(5) $$\begin{array}{c} V\left(\theta \right)=V_{0}E^{\int_{E0}^{\theta }\left[\frac{Gl\text{ Cos}\theta -n}{-\left(1-1\right)Gl\text{ Sin}\theta }\right]\text{d}\theta },\\ \frac{\text{d}y}{\text{d}\theta }=\frac{\text{d}y/\text{d}t}{\text{d}\theta /\text{d}t}=\frac{tV_{0}}{Gt}\frac{{\left(1-\text{Cos}\theta_{0}\right)}^{-2\tau \rho }}{{\left(\text{Sin}\theta_{0}\right)}^{-2\tau \left(1+\rho \right)}}\frac{{\left(\text{Sin}\theta \right)}^{-2\tau \left(1+\rho \right)}\text{Cos}\theta }{{\left(1-\text{Cos}\theta \right)}^{-2\tau \rho }\text{Sin}\theta }. \end{array}$$

In the lunar descent, strategy *τ* consists of a logical impact on several responses for speed with altitude. The variation of altitude determines the fundamental effect. The centrifugal acceleration efficiently adapts the rate of change of the vehicle velocity of vector pitch angle, which impacts the direction of the velocity vector. Hence, the vertical range of the flight path is directly influenced by the term *τ*. By evaluating several values of *τ*, we discover a reasonable count, from which we can then enhance several actions of optimal solutions for speed with altitude.

The article "Hybrid Approach Named HUAPO Technique to Guide the Lander Based on the Landing Trajectory Generation for Unmanned Lunar Mission" was published in 2022. Journal: Comput Intell Neurosci.

### 3.4. Constraints of Lunar Landing

The constraints of lunar landing missions comprise the boundary constraint, which is expressed as follows:

#### 3.4.1. Boundary Constraints

It contains the stages of initial and terminal. Basically, in the lunar missions, the initial stages signify the initial position that is expressed in (6), initial velocity expressed in (7), initial mass exhibited in (8), and initial attitude stated in (9), based on the initial time t0, as follows:

(6) $$\begin{array}{c} R\left(T_{\theta }\right)=r_{\text{Moon}}+H_{0},X\left(T_{0}\right)=X_{0},\beta \left(T_{0}\right)=\beta_{0}. \end{array}$$

(7) $$\begin{array}{c} v_{X}\left(T_{\theta }\right)=v_{X,0,}v_{Y}\left(T_{0}\right)=v_{Y0},v_{Z}\left(T_{0}\right)=v_{Z0}. \end{array}$$

(8) $$\begin{array}{c} M\left(T_{0}\right)=M_{0}. \end{array}$$

(9) $$\begin{array}{c} \varphi \left(T_{0}\right)=\phi_{0}. \end{array}$$

The initial stages signify the orbital elements in (10), the initial mass exhibited in (11), and the initial attitude expressed in (12).

(10) $$\begin{array}{c} v_{X}\left(T_{\theta }\right)=v_{X,0,}v_{Y}\left(T_{0}\right)=v_{Y0},v_{Z}\left(T_{0}\right)=v_{Z0}. \end{array}$$

### 3.5. Trajectory Space Generation

To formulate a focusing flight path developing method as a function of horizontal span and vertical range by using this value of *τ* = 2, all the equations for state variables can be re-extracted. Let *d*_*0*_ and *y*_*0*_ be the first horizontal span and the entire flight path vertical range, and *dt* and *yt* are the terminal values of these parameters. The overall displacements in the horizontal and vertical directions are described as follows:

(11) $$\begin{array}{c} \delta \;D=D_{T}-D_{0}=\sum_{I=1}^{N}\delta D_{i}. \end{array}$$

(12) $$\begin{array}{c} \delta Y=Y_{T}-Y_{0}=\sum_{I=1}^{N}\delta Y_{i}. \end{array}$$

The following section shows the proposed method of the human urbanization algorithm (HUA) and political optimizer (PO) algorithm, as shown in Figure 3. Here, the HUAPO method is employed to handle the thrust fluctuations, checkpoint constraints are suggested for connecting multi-landing phases, angular approach rate is structured to obtain radical change rid, angular approach rate is structured to obtain radical change rid, and safeguards are enforced to deflect collision along with obstacles. Additionally, the problem is first solved based on the proposed HUAPO model.

## 4. Proposed Methodology of Human Urbanization Algorithm (HUA) and Political Optimizer (PO) Algorithm with Radial Basis Functional Neural Network (RBFNN)

In this manuscript, the hybrid approaches of the human urbanization algorithm (HUA) and political optimizer (PO) algorithm with radial basis functional neural network (RBFNN) are proposed; hence, it is named as HUA-PORFNN method. The HUA is a metaheuristic method used to deal with several issues, and several nature-inspired methods have been configured to enhance the convergence speed with quality. PO is motivated by the multiple-phased politics method. The mission's primary purpose is to guide the lander with the lowest fuel consumption from the initial to the final stage, thus minimizing the fuel lunar soft landing issues based on the given cost operation. The TO is categorized as problems arising from disconnection thrust, multiple phase connections, a jump of attitude angle, and avoidance of obstacles. Two main missions of Apollo are (i) Landing from low lunar orbit and (ii) Vertical Takeoff Vertical Landing on the lunar surface. Here, the HUAPO method is implemented to overcome thrust discontinuities, checkpoint constraints are suggested for connecting multi-landing phases, angular approach rate is structured to obtain radical change rid, and safeguards are enforced to deflect collision along with obstacles. Additionally, the problem is solved based on the proposed HUA-PORFNN model. The step-by-step process of the HUA-PORFNN method is shown in Figure 4 and expressed as follows.

The article "Hybrid Approach Named HUAPO Technique to Guide the Lander Based on the Landing Trajectory Generation for Unmanned Lunar Mission" was published in 2022. Journal: Comput Intell Neurosci.

### 4.1. Human Urbanization Algorithm

**Step 1 .**

First, adventurers search for appropriate locations to modify city centers. The equations for adventurers are expressed as follows.

(13) $$\begin{array}{c} x_{i}\left(T\right)=\left(x_{i}^{1},x_{i}^{2},\ldots .x_{i}^{n}\right),i=1,2,\ldots m. \end{array}$$

From the above equation, several adventurers are expressed as *m*, the attribute of the issues is expressed as *n*, and the adventurer, *i* in iteration *t*, is expressed as *Xi(t)*.

The adventurers are updated in each iteration based on the following equation:

(14) $$\begin{array}{c} x_{i}\left(T+1\right)=\frac{k*r*x_{i}\left(T\right)+r*XpR}{k+1}r=1-r. \end{array}$$

Here, *r* denotes a random number of [0, 1]*, XpR* denotes current capital that exhibits the adventurer's experience, and *k* implies the method's parameter to regulate the adventurer's diversification with intensification.

**Step 2 .**

In this step, the adventurers are assessed and have updated the population of cities: (i) in terms of FF, the adventurers are sorted from best to worst, and (ii) every point is evaluated to verify if it is placed on the boundaries of the cities. The updated population of cities is equated based on the following equation:

(15) $$\begin{array}{c} {\text{pop}}_{j}\left(T+1\right)={\text{pop}}_{j}\left(T\right)+{\text{ind}}_{j}. \end{array}$$

From the above equation, the index of city *j* is expressed as *and j*.

The article "Hybrid Approach Named HUAPO Technique to Guide the Lander Based on the Landing Trajectory Generation for Unmanned Lunar Mission" was published in 2022. Journal: Comput Intell Neurosci.

In the form of a circle, the city boundaries can be described. In the circular boundaries of city *j*, the adventure *xi* is situated.

(16) $$\begin{array}{c} \sqrt{{\left(x_{i}^{1}-cNT_{j}^{1}\right)}^{2}+{\left(x_{i}^{2}-cNT_{j}^{2}\right)}^{2}+\cdots +{\left(x_{i}^{n}-cNT_{j}^{n}\right)}^{2}}\leq \text{rad }j. \end{array}$$

Indeed, in the boundaries of squareness, the contribution among the city center vector and adventurer's vector is lesser than the radius of the city.

(17) $$\begin{array}{c} \left|cNT_{j}^{K}-x_{i}^{K}\right|\leq \text{ rad }j,K=1,2,\ldots ,n,\\ \left|cNT_{j}^{K}-x_{i}^{K}\right|\leq \;rad_{j}^{K},K=1,2,\ldots ,n. \end{array}$$

**Step 3 .**

According to the current city centers and points of new adventurers' the novel city center has been chosen. The set of previous city centers with points of adventurers is classified depending upon the fitness function, and the initial *m* points have been selected as novel city centers. Moreover, the center of the first city denotes the capital.

**Step 4 .**

In this step, each city radius is calculated:

(18) $$\begin{array}{c} \text{rad }j\;=\frac{k*\text{diff}*r}{{\text{pop}}_{j}}. \end{array}$$

From the above equation, the radius of city *j* is expressed as *Rad j*, the random number is denoted as *r*, and the population of city *j* is expressed as *Pop j*. Then, depending upon the city center quality, the factor Diff is calculated and compared to the capital-based (19). Directing the search operation to the positive city boundaries is the main objective for connecting the factor *Diff*.

(19) $$\begin{array}{c} \text{Diff}=\text{ARCT }an\left(\left|\frac{\left(f\left(\text{capital}\right)-f\left(cNT_{j}\right)\right)}{f\left(\text{capital}\right)}\right|\right)+0.5. \end{array}$$

(20) $$\begin{array}{c} k=\frac{\left(50*\left(\text{Cos}\left(I*S\right)+1\right)\right)}{I^{rimpK}}, \end{array}$$

From the above equations, the number of iterations is expressed as Itr. Rimpk is another parameter of the method, and in searching the cities' boundaries, it is also utilized for establishing a balance between diversification and intensification. For large values, diversification would be more drastic.

Based on the given equation, to the population of the city, the default value is described.

(21) $$\begin{array}{c} {\text{pop}}_{K}=m-k,K=1,2,\ldots .m. \end{array}$$

According to each city's population, randomly, the populations are spread. Based on the following equation, each citizen place is described as follows:

(22) $$\begin{array}{c} {\text{citizen}}_{j}^{i}=cNT_{j}+\left(r^{i}*{\text{rad}}_{j}\right),i=1,2,\ldots ,{\text{pop}}_{j}j=1,2,\ldots m. \end{array}$$

Here, citizen *j* signifies citizen *i* position of city *j*, and a random number from [−1, 1] is denoted as *Ri.*

The article "Hybrid Approach Named HUAPO Technique to Guide the Lander Based on the Landing Trajectory Generation for Unmanned Lunar Mission" was published in 2022. Journal: Comput Intell Neurosci.

**Step 5 .**

In this step, the city center of each city has the best citizen selected. Then, every center is classified and has finally updated the capital.

At the final stage, the final stage is assessed. If not fulfilled, repeat steps 1 to 5.

### 4.2. Political Optimizer with RBFNN

#### 4.2.1. Prediction of Controller Gain Parameters Using RBFNN

The radial basis factor is considered the activation function for the mathematical modeling of RBFNN. The starting layer is called an input layer used to feed the input data. The network layer is the second layer, also represented as a hidden layer. With the help of radial functions, the network layer is generated. The number of transformations is used between the input layer and network layer. The final layer is called an output layer. A linear combination of radial basis functions of the inputs and neuron parameters is presented in the output layer. The RBFNN is trained by the corresponding values of input and output. The structure, including the training procedure of RBFNN, is depicted as follows. The step-by-step process of RBFNN is expressed as follows:

**Step 6 .**

The Input Vector

The input vector *as* is used in the input layer of the network. Based on the proposed method, the network's input is the time interval *T*; the network output is load demand. The input vector equation is

(23) $$\begin{array}{c} A={\left[A_{1}A_{2}\cdots A_{p}\right]}^{t}, \end{array}$$

where the input vectors of the RBFNN *a* are represented.

**Step 7 .**

The RBF Neurons

Every RBF neuron stores a prototype vector from the training set. All RBF neuron relates their input vector to its prototype. The output becomes in the range of 0 to 1, which is the calculation of equality. When the input is similar to the prototype, the output becomes 1. The activation value is defined as the response value. The prototype vector is defined as the neuron's “center.”

**Step 8 .**

The Output Nodes

The network output contains a set of nodes. All output nodes calculate the score sort to the corresponding group. A classification decision is generally carried out by allocating the input to the group with the most incredible score. From each radial basis function neuron, the score is computed by taking the weighted sum of the activation values. In every radial basis function neuron, an output node connects the weight value to the sum of the weighted. This multiplies the neuron's activity by this weight before adding to the total response. Each output node contains its weights for various groups because every output node calculates the score. Output node presents +ve weight to the radial basis function neurons, and −ve weight is shared with the others.

The article "Hybrid Approach Named HUAPO Technique to Guide the Lander Based on the Landing Trajectory Generation for Unmanned Lunar Mission" was published in 2022. Journal: Comput Intell Neurosci.

**Step 9 .**

Radial Basis Function Neuron Activation Operation

Every radial basis function calculates similarity measures amid the input and prototype vector. Input vectors are identical to the prototype that gives an outcome near 1. Depending on Gaussian, there are various feasible options for similarity functions. The expression of Gaussian including one-dimensional input is

(24) $$\begin{array}{c} F\left(A\right)=\frac{1}{\alpha \sqrt{2\pi }}E^{-\frac{{\left(a-\beta \right)}^{2}}{2\alpha^{2}}}, \end{array}$$

where *a* implies input, *β* implies mean, and *α* implies standard deviation. The radial basis function neuron activation operation is a little different that is expressed as follows:

(25) $$\begin{array}{c} \psi \left(A\right)=E^{-\eta \left\|a-\beta \right\|2}. \end{array}$$

From the above equation, in the Gaussian distribution, *β* is the mean of the distribution.

After completing the algorithm, the RBFNN is efficient in forecasting controller gain parameters as well as generates a combination of optimal solutions based on input time intervals.

**Step 10 .**

Updation

Update the process of the PO algorithm after training and testing.

**Step 11 .**

Party Formation

A political party is generated by individuals with common agenda. The individuals are known as politicians or candidates for public office.

**Step 12 .**

Party Switching

Members can change their affiliation with a party at any time, and a member changing from P1 to P2, P2 to P3, and P3 to P1.  Figure 5 shows the structure of the political optimizer.

**Step 13 .**

Ticket Allocation

From a constituency, the party tickets are allotted to members for the competition of an election. The constituency is deemed a category of voters (constituents) who elect a candidate representing a political party.

**Step 14 .**

Election Campaign

Candidates go to their constituencies and convince their voters to elect them, renewing the candidate's status.

**Step 15 .**

Inter-Party Election

In every constituency, the people vote for a candidate to select a winner.

**Step 16 .**

Government Formation and Parliamentary Affairs

In the parliament, the winners of every candidate are co-ordinates for each other to run the government.

## 5. Result and Discussion

This section presents the result and discussion for the landing trajectory generation of unmanned lunar mission. The mission's primary purpose is to guide the lander with the lowest fuel consumption from the initial to the final stage, thus minimizing the fuel lunar soft landing issues based on the given cost operation. Here, HUAPO method is implemented to deal with the discontinuities of thrust, checkpoint constraints are introduced to connect multiple landing phases, angular attitude rate is designed to get rid of radical changes, and safeguards are enforced to deflect collision with obstacles. Moreover, first, the issues are resolved according to the proposed HUAPO method. Energy trajectories with three different terminal conditions are considered. Additionally, the implementation of the proposed HUAPO method is evaluated in MATLAB/Simulink platform, and the performance of the proposed method is compared with other methods.

The article "Hybrid Approach Named HUAPO Technique to Guide the Lander Based on the Landing Trajectory Generation for Unmanned Lunar Mission" was published in 2022. Journal: Comput Intell Neurosci.

Figure 6 shows the optimized landing trajectories of proposed and reference of altitude, longitude, and latitude. In subplot (a), the optimized landing trajectories of proposed and reference of altitude are presented. Here, the proposed HUA-PORFNN flows at the time period of 450 sec and the altitude is at 15000 m. Then, the reference flows at the time period of 700 sec and the altitude is at 15000 m. Compared to the reference, the simulation time period proposed is low. Subplot (b) presents the optimized landing trajectories of proposed and reference of longitude. Here, the proposed HUA-PORFNN flows at the time period of 310 sec and the longitude is at −1 deg. Then, the reference flows at the time period of 700 sec and the longitude is at −1 deg. Compared to the reference, the simulation time period proposed is low. Subplot (c) presents the optimized landing trajectories of proposed and the reference of latitude. Here, the proposed HUA-PORFNN flows at the time period of 400 sec and the latitude is at −8.8 deg. Then, the reference flows at the time period of 650 sec and the longitude is at −8.8 deg. Compared to the reference, the simulation time period proposed is low.

Figures 6 and 7 show the optimized landing trajectories of proposed and reference of velocity Vx, velocity Vy, and velocity Vz. In subplot (a), the optimized landing trajectories of proposed and reference of altitude are presented. Here, the proposed HUA-PORFNN flows at the time period of 400 sec and the velocity Vx is at −10 m/s. Then, the reference flows at the time period of 650 sec and the velocity Vx is at 0.9 m/s. Subplot (b) presents the optimized landing trajectories of proposed and the reference of velocity Vy. Here, the proposed HUA-PORFNN flows at the time period of 400 sec and the velocity Vy is at 1800 m/s. Then, the reference flows at the time period of 700 sec and the velocity Vy flows at 1800 m/s. Compared to the reference, the simulation time period proposed is low. Subplot (c) presents the optimized landing trajectories of proposed and the reference of velocity Vz. Here, the proposed HUA-PORFNN flows at the time period of 400 sec and the velocity Vz is at 380 m/s. Then, the reference flows at the time period of 650 sec and the velocity Vz is at 380 m/s. Compared to the reference, the simulation time period proposed is low.  Figure 8 shows the optimized landing trajectories of proposed, and reference of pitch, yaw, and thrust is presented.

The article "Hybrid Approach Named HUAPO Technique to Guide the Lander Based on the Landing Trajectory Generation for Unmanned Lunar Mission" was published in 2022. Journal: Comput Intell Neurosci.

In subplot (a), the proposed optimized landing trajectories and pitch reference are presented. Here, the proposed HUA-PORFNN flows at the time period of 12 sec, and the pitch flows at 20 deg. Then, the reference remains constant at 0 deg till the end of the operation. Next, in subplot (b), the optimized landing trajectories of proposed and reference of yaw are presented. Here, the proposed HUA-PORFNN flows at the time period of 400 sec, and the yaw flows at 15 deg. Then, the reference flows at the time period of 700 sec and the yaw flows at −10. Compared to the reference, the simulation time period proposed is low. Finally, in subplot (c), the proposed optimized landing trajectories and the thrust reference are presented.

Here, the proposed HUA-PORFNN flows at the time period of 400 sec and the thrust is at 4.5 N. Then, the reference remains constant at 4.5 N till the end of the operation. Figures 9–11 show the optimized landing trajectories of proposed and reference of altitude, longitude, and latitude. In subplot (a), the optimized landing trajectories of proposed and reference of altitude are presented. Here, the proposed HUA-PORFNN flows at the time period of 450 sec and the altitude is at 15000 m. Then, the reference flows at the time period of 700 sec and the altitude is at 15000 m. Compared to the reference, the simulation time period proposed is low. Subplot (b) presents the optimized landing trajectories of proposed and reference of longitude. Here, the proposed HUA-PORFNN flows at the time period of 310 sec and the longitude is at −1 deg. Then, the reference flows at the time period of 700 sec and the longitude is at −1 deg. Compared to the reference, the simulation time period proposed is low. Subplot (c) presents the optimized landing trajectories of proposed and the reference of latitude. Here, the proposed HUA-PORFNN flows at the time period of 400 sec and the latitude is at −8.8 deg. Then, the reference flows at the time period of 650 sec and the longitude is at −8.8 deg. Compared to the reference, the simulation time period proposed is low.

Figure 10 shows the optimized landing trajectories of proposed and reference velocity Vx, velocity Vy, and velocity Vz. In subplot (a), the optimized landing trajectories of proposed and reference of altitude are presented. Here, the proposed HUA-PORFNN flows at the time period of 400 sec and the velocity Vx is at −10 m/s. Then, the reference flows at the time period of 650 sec and the velocity Vx is at 0.9 m/s. Subplot (b) presents the optimized landing trajectories of proposed and the reference of velocity Vy. Here, the proposed HUA-PORFNN flows at the time period of 400 sec and the velocity Vy is at 1800 m/s. Then, the reference flows at the period of 700 sec and the velocity Vy flows at 1800 m/s. When compared to the reference, the simulation time period proposed is low. Subplot (c) presents the optimized landing trajectories of proposed and the reference of velocity Vz. Here, the proposed HUA-PORFNN flows at the time period of 400 sec and the velocity Vz is at 380 m/s. Then, the reference flows at the time period of 650 sec and the velocity Vz is at 380 m/s. When compared to the reference, the simulation time period proposed is low.  Figure 11 shows the optimized landing trajectories of proposed and reference of pitch, yaw, and thrust. Subplot (a) displays the optimized landing trajectories of the proposed and reference of the pitch. Here, the proposed HUA-PORFNN flows at 12 sec, and the pitch flows at 20 deg. Then, the reference remains constant at 0 deg till the end of the operation. Subplot (b) shows the optimized landing trajectories of proposed and reference of yaw. Here, the proposed HUA-PORFNN flows at the time period of 400 sec, and the yaw flows at 15 deg. Then, the reference flows at the time period of 700 sec and the yaw flows at −10. Compared to the reference, the simulation time period proposed is low. Subplot (c) presents the optimized landing trajectories of proposed and reference of the thrust. Here, the proposed HUA-PORFNN flows at the time period of 400 sec and the thrust is at 4.5 N. Then, the reference remains constant at 4.5 N till the end of the operation.  Figure 12 shows the optimized landing trajectories of proposed and reference of altitude, longitude, and latitude. In subplot (a), the optimized landing trajectories of proposed and reference of altitude are presented. Here, the proposed HUA-PORFNN flows at the time period of 450 sec and the altitude is at 15000 m. Then, the reference flows at the time period of 700 sec and the altitude is at 15000 m. Compared to the reference, the simulation time period proposed is low. Subplot (b) presents the optimized landing trajectories of proposed and reference of longitude. Here, the proposed HUA-PORFNN flows at the time period of 310 sec and the longitude is at −1 deg. Then, the reference flows at the time period of 700 sec and the longitude is at −1 deg. Compared to the reference, the simulation time period proposed is low. Subplot (c) presents the optimized landing trajectories of proposed and the reference of latitude. Here, the proposed HUA-PORFNN flows at the time period of 400 sec and the latitude is at −8.8 deg. Then, the reference flows at the time period of 650 sec and the longitude is at −8.8 deg. Compared to the reference, the simulation time period proposed is low.  Figure 13 shows the optimized landing trajectories of proposed and reference of velocity Vx, velocity Vy, and velocity Vz. In subplot (a), the optimized landing trajectories of proposed and reference of altitude are presented. Here, the proposed HUA-PORFNN flows at the time period of 400 sec and the velocity Vx is at −10 m/s. Then, the reference flows at the time period of 650 sec and the velocity Vx is at 0.9m/s. Subplot (b) presents the optimized landing trajectories of proposed and the reference of velocity Vy. Here, the proposed HUA-PORFNN flows at the time period of 400 sec and the velocity Vy is at 1800 m/s. Then, the reference flows at the time period of 700 sec and the velocity Vy flows at 1800 m/s. Compared to the reference, the simulation time period proposed is low. Subplot (c) presents the optimized landing trajectories of proposed and the reference of velocity Vz. Here, the proposed HUA-PORFNN flows at the time period of 400 sec and the velocity Vz is at 380 m/s. Then, the reference flows at the time period of 650 sec and the velocity Vz is at 380 m/s. Compared to the reference, the simulation time period proposed is low.  Figure 14 shows the optimized landing trajectories of proposed, and reference of pitch, yaw, and thrust is presented. In subplot (a), the proposed optimized landing trajectories and pitch reference are presented. Here, the proposed HUA-PORFNN flows at the time period of 12 sec, and the pitch flows at 20 deg. Then, the reference remains constant at 0 deg till the end of the operation. In subplot (b), the optimized landing trajectories of proposed and reference of yaw are presented. Here, the proposed HUA-PORFNN flows at the time period of 400 sec, and the yaw flows at 15 deg. Then, the reference flows at the time period of 700 sec and the yaw flows at −10. Compared to the reference, the simulation time period proposed is low. Subplot (c) presents the optimized landing trajectories of proposed and reference of the thrust. Here, the proposed HUA-PORFNN flows at the time period of 400 sec and the thrust is at 4.5 N. Then, the reference remains constant at 4.5 N till the end of the operation.

The article "Hybrid Approach Named HUAPO Technique to Guide the Lander Based on the Landing Trajectory Generation for Unmanned Lunar Mission" was published in 2022. Journal: Comput Intell Neurosci.

Table 1 shows the bounds on variables with minimum and maximum values.

Table 2 shows the efficiency of proposed and existing methods.

## 6. Conclusion

This manuscript proposes a hybrid method for landing trajectory generation of unmanned lunar mission. The proposed hybrid control scheme is the joint execution of the human urbanization algorithm (HUA) and political optimizer (PO) with radial basis functional neural network (RBFNN). Hence, it is named as HUA-PORFNN method. The HUA is a metaheuristic method, and it is used to solve several optimization issues and several nature-inspired methods to enhance the convergence speed with quality. On the other hand, multiple-phased political processes inspire the PO. The mission's primary purpose is to guide the lander with the lowest fuel consumption from the initial stage to the final stage, thus minimizing the fuel lunar soft landing issues based on the given cost operation. Here, the HUAPO method is implemented to overcome thrust discontinuities, checkpoint constraints are suggested for connecting multi-landing phases, angular attitude rate is modeled to obtain radical change rid, and safeguards are enforced to deflect collision along with obstacles.

Moreover, first, the issues have been resolved according to the proposed HUAPO method. Here, energy trajectories with 3 terminal processes are deemed. Additionally, the proposed HUAPO method is executed on MATLAB/Simulink site, and the performance of the proposed method is compared with other methods. The lunar landing problem is solved optimally by utilizing the HUAPO method. Using the proposed hybrid method, the system provides an optimal solution with less computation time.

## Figures and Tables

**Figure 1:** Overview of landing lunar mission with proposed method.

**Figure 2:** Structure of lunar mission.

**Figure 3:** Starting and ending stage of the lunar mission.

**Figure 4:** Flowchart of PORFNN.

**Figure 5:** Structure of political optimizer.

**Figure 6:** Optimized landing trajectories of proposed and reference: (a) altitude (b), longitude, (c) latitude.

**Figure 7:** Optimized landing trajectories of proposed and reference: (a) velocity Vx, (b) velocity Vy, (c) latitude Vz.

**Figure 8:** Optimized landing trajectories of proposed and reference: (a) pitch, (b) yaw, (c) thrust.

**Figure 9:** Optimized landing trajectories of proposed and reference: (a) altitude, (b) longitude, (c) latitude.

**Figure 10:** Optimized landing trajectories of proposed and reference: (a) velocity Vx, (b) velocity Vy, (c) latitude Vz.

**Figure 11:** Optimized landing trajectories of proposed and reference: (a) pitch, (b) yaw, (c) thrust.

**Figure 12:** Optimized landing trajectories of proposed and reference: (a) altitude, (b) longitude, (c) latitude.

The article "Hybrid Approach Named HUAPO Technique to Guide the Lander Based on the Landing Trajectory Generation for Unmanned Lunar Mission" was published in 2022. Journal: Comput Intell Neurosci.

**Figure 13:** Optimized landing trajectories of proposed and reference: (a) velocity Vx, (b) velocity Vy, (c) latitude Vz.

**Figure 14:** Optimized landing trajectories of proposed and reference: (a) pitch, (b) yaw, (c) thrust.

**Table 1:** Bounds of variables.

Variables	Min	Max	Variable	Min	Max
*H*	0	30 km	*ωφ*	-8/s	8/s
*φ*	−20	90	*ωψ*	-8/s	8/s
*ψ*	−180	180	T	4671 N	43148 N

**Table 2:** Efficiency of proposed and existing methods.

Solution technique	Efficiency (%)
HUA-PORFNN	95.18
Reference	92.57

## Data Availability

All required data are available in the article.
